The article "CD3+T, CD4+T, CD8+T, and CD4+T/CD8+T Ratio and Quantity of γδT Cells in Peripheral Blood of HIV-Infected/AIDS Patients and Its Clinical Significance" was retracted in 2023. Reasons: unreliable results or conclusions; concerns about the data; concerns about the peer review; concerns about the citations.

# CD3^+^T, CD4^+^T, CD8^+^T, and CD4^+^T/CD8^+^T Ratio and Quantity of *γδ*T Cells in Peripheral Blood of HIV-Infected/AIDS Patients and Its Clinical Significance

**DOI:** 10.1155/2021/8746264

**Published:** 2021-12-08

**Authors:** Nange Zhao, Tingting Zhang, Yujuan Zhao, Jianping Zhang, Keqiang Wang

**Affiliations:** ^1^Department of Laboratory Medicine, Second Affiliated Hospital of Shandong First Medical University, Taian City 271000, Shandong Province, China; ^2^Department of Laboratory Medicine, Xianyang Central Hospital, Xianyang City, 712000 Shanxi Province, China; ^3^Department of Emergency Medicine, Yingsheng District, Tai'an Central Hospital, Taian City 271000, Shandong Province, China

## Abstract

**Objective:**

To investigate the quantity of CD4^+^T, CD4^+^T, CD8^+^T, and *γδ*T cells in peripheral blood of HIV-infected/AIDS patients as well as to explore the possible role of CD4/CD8 ratio and *γδ*T cells in the progression of HIV/AIDS, aimed at providing evidence for the diagnosis and treatment of AIDS.

**Methods:**

The quantity levels of CD3^+^T cells, CD4^+^T cells, CD8^+^T cells, and *γδ*T cells in peripheral blood of 46 HIV-infected/AIDS patients and 30 healthy controls were detected by using flow cytometry.

**Results:**

The count of CD3^+^T, CD4^+^T, CD8^+^T, and *γδ*T cells ($\bar{x}\pm s$, A/*μ*l) in the peripheral blood was 1183.64 ± 132.58, 278.39 ± 122.38, 863.13 ± 82.38, and 22.53 ± 1.74 in the experimental group as well as 1456.46 ± 124.37, 788.74 ± 189.67, 569.61 ± 46.49, and 10.96 ± 0.28 in the control group, respectively. The *p* values of the two groups were <0.005 after the *t*-test, revealing a statistically significant difference. The proportion of CD3^+^T, CD4^+^T, CD8^+^T, and *γδ*T cells in total lymphocytes in the two groups ($\bar{x}\pm s$, %) was 71.83 ± 5.37, 13.39 ± 2.23, 62.93 ± 5.81, and 3.67 ± 0.87 in the experimental group, respectively. In the control group, the values were expressed as 66.72 ± 5.48, 42.77 ± 3.38, 31.41 ± 3.62, and 1.73 ± 0.36, respectively. After performing the *t*-test, *p* values in the two groups were <0.005 except CD3^+^T, with statistically significant differences. Besides, CD4/CD8 was 0.33 ± 0.11 in the experimental group and 1.48 ± 0.29 in the control group, *t* = 26.528, *p* < 0.001, exhibiting a significant statistical difference.

**Conclusion:**

HIV infection induces the activation and proliferation of CD8^+^T and *γδ*T cells, contributing to the decrease of CD4^+^T cells, while CD8^+^T and *γδ*T cells are involved in the immune response and tissue damage after HIV infection.

## 1. Introduction

Currently, HIV infection is considered one of the most serious infectious diseases in the world, which mainly causes damage or even defects of immune cells and organism function by infecting and destroying CD4^+^T lymphocytes, eventually being complicated with various serious opportunistic infections and tumors [1]. Although the immunological mechanism of HIV infection in the body (for example, CD4^+^T cell decline) has been partially established, the exact immune regulatory mechanism is unclear. At present, there is no specific treatment, and nonspecific antiviral therapy has become the first attempt [2–5]. Impaired immune function remains a major problem in HIV infection, primarily due to CD4^+^T cell decline and hypofunction, which is attributed to the lytic destruction of infected CD4^+^T lymphocytes by HIV and the damage caused by the targeting of uninfected CD4^+^T cells by the glycoprotein gp120, which is attacked by CD8^+^ cytotoxic T cell-mediated cytotoxicity (CTL) and antibody-dependent cytotoxicity (ADCC). The proportion of CD4^+^T lymphocyte subsets TH1/TH2 is imbalanced, resulting in decreased function [6]. According to different T cell antigen receptors (TCR), T cells are categorized into *αβ*T cells and *γδ*T cells. The latter is composed of *γ* chains and *δ* chains, and the number is relatively small, occupying 0.5%-5% of healthy adult lymphocytes [7–10]. *γδ*T cells originate from the thymus but mature in peripheral tissues and organs. Most of the *γδ*T cells are CD4^−^ and CD8^−^ cells, and a few are CD4^+^ and CD8^+^ cells. In recent years, *γδ*T cells have attracted much attention due to their regulatory function on CD4^+^ and CD8^+^T lymphocytes, their ability to rapidly proliferate after infection, and their ability to directly recognize antigens without antigen presentation [11]. In the present study, by detecting the peripheral blood CD3^+^T, CD4^+^T, CD8^+^T, and *γδ*T cells of HIV-infected/AIDS patients, the number of *γδ*T, CD4^+^T, and CD8^+^T cells and HIV infection in HIV-infected/AIDS patients can be identified. The relationship with disease progression provides a basis for adoptive immunotherapy and other treatment methods for AIDS.

## 2. Materials and Methods

### 2.1. Research Object

In this study, a total of 46 HIV-infected/AIDS patients admitted to a hospital in Xianyang from January 2019 to October 2019 were selected as the experimental group. There were 27 males and 19 females, aged from 19 to 69 years, with an average of 42.59 ± 4.28 years. Besides, thirty healthy subjects who came to the hospital's physical examination center during the same period served as the control group. There were 17 males and 13 females, aged 18 to 65 years, with an average of 43.08 ± 4.19 years.

### 2.2. Standard Constraint

The following are the standard constraints: (1) 15 (inclusive) to 75 (inclusive) years of age, regardless of gender; (2) ELISA and Western blotting methods adopted for detecting the positive HIV-1 antibody, or the positive HIV nucleic acid test; (3) has not received ART treatment previously; (4) subjects having informed consent to the treatment method; (5) diagnostic criteria satisfying the “Diagnostic Criteria for AIDS and HIV Infection (2019 Edition)” (National Health Commission, hereinafter referred to as “Diagnostic Criteria”); and (6) informed consent of patients and their families.

### 2.3. Exclusion Criteria

The exclusion criteria are the following: (1) pregnant and lactating women; (2) special medical history; (3) active opportunistic infection within 2 weeks before enrollment; (4) drug abuse history, which may affect the results of the present study; and (5) poor compliance of subjects.

### 2.4. Main Reagents and Equipment

The main reagents and equipment are (1) monoclonal antibodies: CD3/CD4/CD8/CD45 four-color antibody (product number: 561707), CD3APC (product number: 30062), CD4PerCP (product number: 100538), CD3-FITC/CD8-PE/CD4-APC (product number: 561644), and *γδ*TCR APC (product number: 561995) (produced by Becton Dickinson, USA); (2) FACSCalibur flow cytometer (produced by Becton Dickinson, USA); (3) EDTA-K2 anticoagulant vacuum blood collection tube (produced by Becton Dickinson, USA); (4) microplate reader (RT-6100, produced by Rayto, USA); and (5) centrifuge (produced by Eppendorf, Germany, type 5424R).

### 2.5. Specimen Collection

The specimen collection procedure is as follows: (1) Collect 2 ml of the subject's peripheral venous blood on an empty stomach in the morning, place it in an EDTA anticoagulation tube, and mix it well. (2) Take 2 ml of the abovementioned venous whole blood and then test it within 3 hours.

### 2.6. Determination of Absolute Counts and Percentages of CD3^+^T, CD4^+^T, and CD8^+^T Lymphocytes

(1) Take one absolute counting tube from each specimen and add 20*μ*l of CD3/CD4/CD8/CD45 four-color antibodies, namely, CD3-FITC fluorescent-labeled antibodies, CD8-PE fluorescent-labeled antibodies, CD4-PreCP, and CD4-APC fluorescent-labeled antibodies; (2) add 100 *μ*l of whole blood to each, followed by mixing gently and storing in the dark at room temperature for 15 minutes; (3) supplement 1 to each tube × FACS Lysing Solution 2 ml; (4) mix evenly lysed red blood cells and place them in the dark at room temperature for 10 min; (5) centrifuge at 1000 r/min for 5 min, wash, add 500 *μ*l PBS for mixing, and place for 5 min; (6 ) perform upflow cytometer detection, after power on, automatically check the instrument by FACScomp software; set the experimental acquisition conditions such as the voltage, photomultiplier tube and fluorescence compensation; employ MultiSET automatic analysis software to obtain the number of T lymphocytes (CD3^+^); analyze and record CD3^+^, the absolute count of CD4^+^CD8^−^ T cells, the absolute count of CD3^+^ CD4^−^CD8^+^T cells, and the percentage of both of them in lymphocytes and CD3^+^.

### 2.7. Determination of the Absolute Count and Percentage of *γδ*T Cells

For determination of the absolute count and percentage of *γδ*T cells, (1) take the control tube and the measurement tube and add 20 *μ*l each of CD3 and *γδ*TCR antibodies; (2) add 50 *μ*l of whole blood, gently shake and mix, and place at room temperature away from light for 15 minutes (3) supplement 1 ml 1×FACS Lysing Solution to each tube, gently shake and mix, and place in the dark at room temperature for 10 min; (4) centrifuge at 1000 r/min for 5 min, wash, and add 500 *μ*l PBS; for resuspending; (5) add 100 *μ*l of fluorescent microspheres; (6) conduct up-flow cytometer detection, after power on, automatically check the instrument, via FACScomp software, calibrate the instrument detection conditions with microspheres, and set the voltage, photomultiplier tube, fluorescence compensation and other experimental acquisition conditions, using Cellquest. The analysis software divides the cell population by forward scattered light and side scattered light, and obtains the number of T lymphocytes (CD3^+^). After that, taking CD3^+^T lymphocytes as the gate, calculate the absolute value and percentage of *γδ* T cells in the gate.

### 2.8. Statistical Analysis

SPSS23.0 software was employed for performing statistical analysis. Normally distributed measurement data are described by $\bar{x}\pm s$, two samples are compared by the *t*-test, and multiple groups are compared by the *F* test. The difference is statically significant with *p* < 0.05.

## 3. Result

### 3.1. Comparison of the Absolute Counts of CD3^+^T, CD4^+^T, CD8^+^T, and *γδ*T Cells in the Peripheral Blood of the Experimental and Control Groups

The absolute counts of CD3^+^T, CD4^+^T, CD8^+^T, and *γδ*T cells in the peripheral blood of the experimental group and the control group are illustrated in Table 1 and Figure 1. The numbers of CD3^+^T and CD4^+^T cells in the experimental group were lower than those in the control group. Those of CD8^+^T cells and *γδ*T cells were higher than those in the control group. Apart from that, the difference was statistically significant at *p* < 0.05.

### 3.2. The Proportion of CD3^+^T, CD4^+^T, CD8^+^T, and *γδ*T Cells in Lymphocytes in the Experimental and Control Groups

The percentages of CD3^+^T, CD4^+^T, CD8^+^T, and *γδ*T cells in lymphocytes in the experimental group and the control group are displayed in Tables 2 and 3 and Figures 2–5. There existed no significant difference in the proportion of CD3^+^ in total lymphocytes between the two groups (*p* > 0.05). The proportion of CD4^+^T cells in lymphocytes and the ratio of CD4/CD8 in the experimental group were lower compared with those in the control group. In the experimental group, CD8^+^ and the proportion of *γδ*T cells in lymphocytes were higher than that of the control group. The proportions of CD8^+^ and *γδ*T cells in CD3^+^ cells in the experimental group were higher than those in the control group. The proportion of CD4^+^T cells in CD3^+^ cells in the experimental group was lower than that in the control group. In the control group, the differences showed a statistical difference (*p* < 0.05).

## 4. Discuss

### 4.1. CD4^+^T Cells and HIV Infection

CD4^+^T lymphocytes are the central cells of immune response and the main target cells of HIV infection [12, 13]. Among normal people, CD4^+^T lymphocytes account for approximately 65% of the total T lymphocytes. After HIV enters the human body, it first attacks CD4^+^T cells through a variety of ways and methods, generating a decrease in their number, impaired cell function, and abnormal immune activation [14]. In the early stage of HIV infection, the virus replicates efficiently in the lymph nodes, CD4^+^T cells are activated, and the virus proliferates in the cells, leading to cytopathic toxicity, which consequently causes metabolic dysfunction of CD4^+^T cells. Although Th1 cellular immune response can suppress the virus, it fails to eliminate the virus and infected cells. Due to the continuous decrease in the number of CD4^+^T cells and the decrease in the cytokines released by Th1, it causes the failure and defects of the body's cellular immune function, ultimately leading to the proliferation of opportunistic pathogens in the body's tissue system and organs as well as the occurrence of selective tumors. As a result, opportunistic infection and tumors can be generated. In the present study, among the lymphocytes and CD3^+^T cells, the quantity of CD4^+^T cells in HIV-infected/AIDS patients was significantly lower than that in the healthy control group. In addition, the proportion of CD4^+^T cells was significantly lower than that in the control group. The research is in consistence with [15]. It indicates that the immune function of HIV-infected persons/AIDS patients is impaired, and the proportion of CD4^+^T cells in lymphocytes decreases.

The current research on the mechanism of the reduction of CD4^+^T cells caused by HIV infection has not yet formed a unified opinion. Three theories are included including the increase in the destruction of CD4^+^T cells by HIV reducing them, the damage of thymus function caused by HIV, and the presence of T cells. Lymphatic tissue is retained [16]. Most studies consider that the reason for the progressive decrease of CD4^+^T cells after HIV infection may be related to cell apoptosis after HIV infection [17], and it can be employed as an indicator for evaluating the effect of antiviral treatment, which is important for opportunistic infection and death (parameters [18]).

### 4.2. CD8^+^T Cells and HIV Infection

CD8^+^T lymphocytes are the effector cells of specific cellular immunity. Normal people account for approximately 35% of the total T lymphocytes. They can specifically identify the target cells infected by the virus to dominate a killing effect on the virus. It is the body's ability to kill HIV. Main immune cells exert direct killing effect [19]. The mechanism of its action on HIV includes the following: (1) direct killing effect: cells infected by HIV are directly killed by perforin (perforin) and granzyme B (granzyme B), and target cell apoptosis is induced by CD95L (Fas Ligand), aimed at eliminating the infectious agent; (2) inhibit virus replication: inhibit virus replication by producing cytokines such as interferon C; (3) release MIP-1A, MIP-1B, and other chemokines to block the virus from entering new target cells. In the current work, different from the results of CD4^+^T cells, the quantity of CD8^+^T cells in white blood cells, lymphocytes, and CD3^+^ cells was significantly higher than that of the healthy control group, and the proportion was obviously higher than that of the control group. Additionally, it demonstrates that with the continuous replication of HIV in the body, the body's immune cell function is impaired, CD4^+^ cells decrease, and CD8^+^ cells increase accordingly.

### 4.3. CD4/CD8 Ratio and HIV Infection

In the peripheral blood of normal people, the ratio of CD4/CD8 is 1.5 to 2.0. After HIV infects the body, regardless of whether the patient has clinical symptoms, there will exist a decline in CD4^+^T lymphocytes. The decline is even greater in patients undergoing tumors and opportunistic infections. When the course of the disease progresses, CD8^+^T cells will decrease as the absolute lymphocyte count decreases. In the terminal stage of the disease, the remaining lymphocytes in the body are almost all CD8^+^T cells. In other stages other than the terminal stage of the disease, CD8^+^T cells will increase, contributing to an inversion of the CD4/CD8 ratio [20]. In the present study, the CD4/CD8 ratios of HIV-infected persons/AIDS patients were lower than those of the control group, and the difference was statistically significant (*p* < 0.05). It is consistent with the research of Lin [21]. It is suggested that the ratio of CD4/CD8 can reflect the damage of immune function in HIV-infected/AIDS patients. There are data reports that the absolute counts of lymphocytes and their subgroups are easily affected by drugs, race, viral infections, etc., while the ratio between T lymphocyte subgroups remains comparatively stable. As a result, compared with the CD4^+^T cell count, the CD4/CD8 ratio is more stable in judging HIV-infected persons/AIDS patients and provides greater significance [22]. The CD4/CD8 ratio is positively correlated with CD4^+^ levels, which is negatively correlated with viral load [23]. It is often used clinically to reflect the status of HIV disease as one of the important indicators of disease progression. Additionally, the CD4/CD8 ratio can also provide HIV-infected/AIDS patients with the same prognostic information as the CD4 cell count, which can also be used as a predictor of the prognosis of AIDS patients.

### 4.4. *γδ*T Cells and HIV Infection

*γδ*T cells are a group of special T cells that express *γ* and *δ* chains. They are the body's innate immune cells and an important component involved in natural immunity. Besides, they are mainly distributed in mucosa and subcutaneous tissues, such as the small intestine, skin and lungs, and epidermis and membrane tissue epithelium. Besides, it is one of the main components of internal lymphocytes [11, 24]. Recent studies have shown that *γδ*T cells play an important role in antitumor, anti-infection, and immune regulation [25–31]. In human peripheral blood, TCR*γδ* accounts for approximately 0.5%-5%, mainly expressed on the surface of CD3^+^T cells, and participates in the regulation of various physiological functions of the human body, containing immune regulation, immune protection, immune homeostasis, immune killing, inflammation, immune surveillance, autoimmunity, and cytotoxicity. Because *γδ*T cells have regulatory functions on CD4^+^ and CD8^+^T lymphocytes, the ability to rapidly proliferate after infection, and the ability to directly recognize antigens without antigen presentation [11], *γδ*T cells play a pivotal role in the body's mucosal immunity and antivirus. In recent years, its damage in early HIV infection has received attention and is considered to exist an important role in fighting HIV infection. HIV does not directly cause infection damage to *γδ*T cells but can be used as a marker of viral infection and disease progression [32], aimed at regulating mucosal immune infection in HIV-infected patients. The anti-HIV mechanism of *γδ*T cells includes regulating the function of CD8^+^T lymphocytes, exerting a direct killing effect on infected cells, and secreting macrophage inflammatory proteins, CC type chemokine ligand 5, and other chemokines that inhibit viral infection and replication [33]. In addition, it plays an important role in the suppression of the virus by elite controllers of HIV infection.

In the current work, by flow cytometry, *γδ*T cells were highly expressed in HIV-infected/AIDS patients, and the proportion of lymphocytes in HIV-infected/AIDS patients and healthy controls was 27.47 ± 3.52% and 15.73 ± 2.36%, which was similar to the results of Wang et al. [34]. By testing 39 HIV-infected/AIDS patients and 20 healthy subjects, the proportions of *γδ*T cells were 18.1 ± 10.1% and 15.2 ± 8.9%, respectively. After antiviral treatment, the percentage of *γδ*T cells in HIV-infected and AIDS patients was significantly reduced. Meanwhile, the percentage of *αβ*T cells was significantly increased. Therefore, it is suggested that HIV infection can generate the increase of *γδ*T cells and exert their immune killing, immune regulation, and cytotoxic effects.

In summary, HIV infection induces the activation and proliferation of CD8^+^T and *γδ*T cells, which in turn leads to decrease in the number of CD4^+^T cells. CD8^+^T and *γδ*T cells participate in the immune response and tissue damage process caused by HIV infection. The immune function of HIV-infected persons is impaired. The proportion of CD4^+^T cells in lymphocytes decreases. The number of T lymphocytes has a decisive effect on the immune function of the body. When the CD4^+^T cell count decreases, the condition of HIV-infected/AIDS patients will become more serious and the chance of opportunistic infections will accordingly increase. In HIV-infected persons, the absolute count and percentage of CD3^+^T cells are different and abnormal while they are still within the reference interval. This may be due to the steady state compensation of CD8^+^T cell changes in HIV-infected persons. CD4^+^T, CD8^+^T, and *γδ*T cell count can reflect the number of HIV-infected target cells, and its count level can be employed as an important indicator to reflect the immune status of the body, as well as a marker for monitoring the progress of AIDS and judging the condition of patients, which can be used as an evaluation of antivirus. The indicators of treatment effect and the important parameters of opportunistic infection and death provide a significant basis for antiviral treatment. Additionally, the CD4/CD8 ratio can also provide HIV-infected/AIDS patients with the same prognostic information as the CD4 cell count, which can be used as a predictor of the prognosis of AIDS patients.

## Figures and Tables

**Figure 1:** Comparison of absolute counts of CD3^+^T, CD4^+^T, CD8^+^T, and *γδ*T cells in peripheral blood between the two groups. Note: (a–d) are the comparisons of the absolute numbers of CD3^+^T, CD4^+^T, CD8^+^T, and *γδ*T cells in the two groups, respectively.

**Figure 2:** Comparison of the proportion of CD3^+^T, CD4^+^T, CD8^+^T, and *γδ*T cells in total lymphocytes between the two groups. Note: (a–e) are the comparison of the proportions of CD3^+^T, CD4^+^T, CD8^+^T, and *γδ*T cells in the total lymphocytes in the two groups ($\bar{x}\pm s$, %).

**Figure 3:** The proportion of CD3^+^T, CD4^+^T, CD8^+^T, and *γδ*T cells in the total lymphocytes of the experimental group detected by flow cytometry. Note: (a–d) are the percentages of CD3^+^T, CD4^+^T, CD8^+^T, and *γδ*T cells in the total lymphocytes in the experimental group detected by flow cytometry.

**Figure 4:** The proportion of CD3^+^T, CD4^+^T, CD8^+^T, and *γδ*T cells in the total lymphocyte in the control group was detected by flow cytometry. Note: (a–d) are the proportions of CD3^+^T, CD4^+^T, CD8^+^T, and *γδ*T cells in the total lymphocytes in the control group detected by flow cytometry.

**Figure 5:** Comparison of the proportion of CD4^+^T, CD8^+^T, and *γδ*T cells in CD3^+^T cells between the two groups ($\bar{x}\pm s$, %). Note: (a–c) are the comparison of the proportions of CD4^+^T, CD8^+^T, and *γδ*T cells in CD3^+^T cells between the two groups ($\bar{x}\pm s$, %).

**Table 1:** Comparison of absolute counts of CD3^+^T, CD4^+^T, CD8^+^T cells, and *γδ*T cells between the two groups ($\bar{x}\pm s$, A/*μ*l).

Group	CD3^+^T	CD4^+^T	CD8^+^T	*γδ*T
Experimental group (46 cases)	1183.64 ± 132.58	278.39 ± 122.38	863.13 ± 82.38	22.53 ± 1.74
Control group (30 cases)	1456.46 ± 124.37	788.74 ± 189.67	569.61 ± 46.49	10.96 ± 0.28
*t*	6.665	14.276	17.735	36.036
*p*	0.003	<0.001	<0.001	<0.001

**Table 2:** The proportion of CD3^+^T, CD4^+^T, CD8^+^T, and *γδ*T cells in total lymphocytes in the two groups ($\bar{x}\pm s$, %).

Group	CD3^+^T	CD4^+^T	CD8^+^T	CD4/CD8	*γδ*T
Experimental group (46 cases)	71.83 ± 5.37	13.39 ± 2.23	62.93 ± 5.81	0.33 ± 0.11	3.67 ± 0.87
Control group (30 cases)	66.72 ± 5.48	42.77 ± 3.38	31.41 ± 3.62	1.48 ± 0.29	1.73 ± 0.36
*t*	1.661	45.711	29.037	26.528	11.564
*p*	0.101	<0.001	<0.001	<0.001	<0.001

**Table 3:** The proportion of CD4^+^T, CD8^+^T, and *γδ*T cells in CD3^+^T cells in the two groups ($\bar{x}\pm s$, %).

Group	CD4^+^T	CD8^+^T	*γδ*T
Experimental group (46 cases)	16.59 ± 2.23	56.89 ± 7.67	5.18 ± 1.27
Control group (30 cases)	59.43 ± 5.27	41.36 ± 5.59	2.54 ± 0.12
*t*	34.884	19.548	11.327
*p*	<0.001	<0.001	<0.001

## Data Availability

The data used to support the findings of this study are available from the corresponding author upon request.
